The article "Efficacy of Periodontal Endodontics Combined with Diode Laser (DL) Therapy on Severe Periodontitis" was retracted in 2023. Reasons: signs of a paper mill; suspected computer-generated content; unreliable results or conclusions; lack of ethics approval or compliance.

# Efficacy of Periodontal Endodontics Combined with Diode Laser (DL) Therapy on Severe Periodontitis

**DOI:** 10.1155/2022/5689900

**Published:** 2022-10-15

**Authors:** Sijia Liu, Xu Zhang, Quanying Zhou

**Affiliations:** ^1^Wuhan Hospital of Traditional Chinese Medicine, Department of Stomatology, No. 303 Sixin Avenue, Hanyang, Wuhan 430000, Hubei, China; ^2^Wuchang Hospital Affiliated to Wuhan University of Science and Technology (Stomatology), No. 116 Yangyuan Street, Wuchang District, Wuhan 430063, Hubei, China; ^3^Wuhan 9th Hospital, Department Stomatology, No. 20, Jilin Street, Qingshan District, Wuhan 430080, Hubei, China

## Abstract

**Background:**

For a long time, the impact of severe periodontitis on the pulp has been the focus of periodontal clinical research. Whether the teeth with severe periodontitis should be treated with pulp has also become the focus of clinical research.

**Aims:**

To explore the effect of periodontal endodontic therapy combined with DL therapy on severe periodontitis.

**Materials and Methods:**

The clinical data of 100 patients with severe periodontitis from January 2020 to July 2022 were selected and included in the retrospective study. According to the different retrieval treatment methods, they were divided into the control group and the treatment group with 50 cases in each group. The control group received periodontal endodontic treatment, and the treatment group received DL treatment on the basis of the control group. The differences in periodontal probing depth (PD), toothache degree, bleeding index (BI), inflammatory factors, plaque index (PLI), and attachment loss (AL) between the two groups were compared and analyzed.

**Results:**

After 3 months of treatment, the bleeding index (BI), plaque index (PLI), and periodontal probing depth (PD) of the treatment group were significantly lower than those of the control group, and the difference was statistically significant (*P* < 0.05). The attachment loss (AL) of the group was not significantly different from that of the control group (*P* > 0.05). Before treatment, there was no significant difference in the levels of inflammatory factors between the two groups (*P* > 0.05). After 3 months of treatment, the levels of IL-6 and CRP in the treatment group were significantly lower than those in the control group, and the difference was statistically significant (*P* < 0.05). Before treatment, there was no significant difference in the levels of inflammatory factors between the two groups (*P* > 0.05). After 3 days of treatment, the VAS score of the treatment group was significantly lower than that of the control group, and the difference was statistically significant (*P* < 0.05).After treatment, there were no complications during follow-up in the two groups.

The article "Efficacy of Periodontal Endodontics Combined with Diode Laser (DL) Therapy on Severe Periodontitis" was retracted in 2023. Reasons: signs of a paper mill; suspected computer-generated content; unreliable results or conclusions; lack of ethics approval or compliance.

**Conclusion:**

The application of DL treatment has a significant effect, which can promote the healing of periodontal tissue, reduce the depth of periodontal pockets, and reduce the degree of toothache, thereby providing a reference for clinical treatment.

## 1. Introduction

Severe periodontitis is one of the difficult aspects of periodontal treatment due to the fact that severe periodontitis not only destroys the periodontal tissue [1], but it also leaves the pulp in a subclinical state through periodontal pulp traffic branches, and the presence of diseased pulp will prevent the healing of periodontal tissue after periodontal treatment [2]. Severe periodontitis is a common disease in dentistry, the onset of which is associated with multiple factors, and early patients have no obvious symptoms, mostly just secondary gingival bleeding or halitosis, with symptoms similar to gingival inflammation [3]. With the development of the disease, patients can develop corresponding symptoms, which affect the chewing function of teeth and reduce the quality of life of patients [4]. Severe periodontitis tends to involve several tissues, while the anatomical structure between periodontal and pulpal tissues is relatively special, involving dentin tubules and apical foramina [5]. The relationship between the two tissues is interoperable, and unilateral lesions and infections may affect the other side, resulting in combined periodontal and pulpal lesions that make treatment more difficult [6].

A large number of studies in recent years have shown the efficacy of periodontal-endodontic treatment of severe periodontitis, which can reduce the depth of periodontal pockets and positively control the disease [7]. However, in view of the limitations of the results achieved by single treatment, it has been suggested that DL can be combined to enhance the therapeutic effect from different mechanisms of action [8]. The principle of action of DL is a treatment that uses mechanical, photochemical, thermal, and biological promotion effects to accelerate the inflammation relief at the lesion site [9]. The laser has a bactericidal effect, especially in periodontal soft tissues, as DL has an affinity for hemoglobin and gingival pigments, allowing precise soft tissue separation, sealing of blood vessels, and removal of the working area, while reducing postoperative swelling [10]. In addition, DL has the advantages of portability, affordability, and ease of operation [11]. DL is more effective and less invasive than traditional methods. DL allows precise cutting of soft tissues and complete debridement of diseased tissues while looking directly at the affected tooth and has the efficacy of removing subgingival plaque and tartar and inhibiting periodontitis pathogens, and it has been widely used in periodontal treatment in recent years [12]. Therefore, in this study, periodontal endodontic treatment combined with DL treatment was performed in patients with severe periodontitis.

The article "Efficacy of Periodontal Endodontics Combined with Diode Laser (DL) Therapy on Severe Periodontitis" was retracted in 2023. Reasons: signs of a paper mill; suspected computer-generated content; unreliable results or conclusions; lack of ethics approval or compliance.

## 2. Material and Methods

### 2.1. Research Object

The clinical data of 100 patients with severe periodontitis from January 2020 to July 2022 were selected for inclusion in the retrospective study. Fifty cases each were divided into a comparison group and a treatment group according to the retrieval treatment method. Diagnostic criteria for periodontitis are as follows [13]: adjacent CAL detected in more than 2 nonadjacent teeth; or the presence of buccal or lingual CAL ≥3 mm in >2 teeth, along with PD ≥ 3 mm.

### 2.2. Criteria for Nadir Discharge

Inclusion criteria are as follows:(i) age 18 to 70 years old, clinical attachment loss ≥5 mm, apical radiograph showing alveolar bone destruction exceeding 1/2 of root length, degree of loosening less than 3 degrees, sluggish pulp viability test, and no clinical pulp tooth with inflammation symptoms; (ii) there is no obvious loosening of the tooth, no full crown restoration, periodontal and endodontic joint disease, or grade III furcation disease; (iii) in order to avoid false negative or false positive results of the electrical measuring instrument at the same time, perform a pulp temperature test on the affected tooth, choose the thermal diagnosis method of gutta-percha, first measure the control tooth, and then measure the test tooth. Sexual pain. Exclusion criteria are as follows: (i) women who are pregnant, breastfeeding, or planning to become pregnant within the past 3 months, patients with acute periodontal abscess or acute necrotizing gingivitis; (ii) history of periodontal treatment within the past 3 months, within the past 3 months history of taking antibiotics, nonhormonal anti-inflammatory drugs and immune preparations, and other systemic diseases; (iii) patients with systemic diseases, smokers, dentin sensitivity, poor restorations, or night grinding.

### 2.3. Methods

The control group was given periodontal endodontic treatment, that is, a comprehensive specialist examination was performed on the patients, detailed medical history and periodontal records were taken, and oral hygiene education was given to the patients, and the test teeth were selected. Full-mouth ultrasonic supragingival scaling was performed first, the clinical indicators of the test teeth were recorded, and a standard series of periapical films were taken. Root canal treatment was performed on the teeth of test group 1 (the criteria for the success of root canal treatment were X-ray that showed the root canal filling was tight, and the root filling was 0.5-2 m away from the apex. Satisfied), one week after treatment, ultrasonic scaler and Gracey subgingival scaling device were used to complete subgingival scaling and root planing in two times.

The article "Efficacy of Periodontal Endodontics Combined with Diode Laser (DL) Therapy on Severe Periodontitis" was retracted in 2023. Reasons: signs of a paper mill; suspected computer-generated content; unreliable results or conclusions; lack of ethics approval or compliance.

The treatment group was combined with DL treatment on the basis of the control group, that is, adjusting the DL display screen to the periodontal scaling, according to the depth of periodontal probing, gently probe the 400 m optical fiber into the bottom of the periodontal pocket, and lift it 2 mm and move it to feel it. Its form. Start the laser (wavelength 980 nm, power 2 W), keep the tip of the fiber in contact with the epithelial tissue, and make a “zigzag” movement in the periodontal pocket smoothly and slowly. When the periodontal pocket is less than 6 mm, the laser irradiation time is about 30 s, and when the periodontal pocket is larger than 6 mm, the irradiation time is 45 s. Routine ultrasonic subgingival scaling and manual root planing were then performed. After the conventional treatment, the laser treatment is used again for about 20∼30 s for the purpose of hemostasis and periodontal debridement.

#### 2.3.1. Observation Indexes

(i) PD: 6 sites (labial-buccal/lingual mesial, central, and distal) were recorded for each tooth, in millimeters (mm), rounded up, and the probing force was controlled at 20-25 g. BI: record both buccal and lingual surfaces for each tooth. The scoring criteria are as follows: 0 is healthy gums without inflammation and bleeding; 1 is inflammatory changes in the color of the gums without bleeding on probing; 2 is punctate bleeding after probing; 3 is bleeding after probing that spreads along the gingival margin; 4 is bleeding that overflows and overflows the gingival sulcus; 5 is spontaneous bleeding. PLI: plaque index scoring method was employed, the buccal and lingual surfaces of each tooth are recorded, and the scoring standard is as follows: 0 is sterile plaque in the gingival margin area and 1 is thin plaque on the tooth surface in the gingival margin area; however, it is not easy to see by visual inspection. The side of the probe tip is used to scrape out plaque. AL: when the gingiva is coronal to the cementoenamel junction, AL is the periodontal probing depth distance from the cementoenamel junction to the gingival margin. (ii) 4 mL of fasting venous blood was extracted from patients for inflammatory factor levels, and after centrifugation at 3000 r/min for 10 min, the supernatant was taken, and the American Beckman Coulter AU-5800 automatic biochemical analyzer was used which was provided by Beijing Hotgen Biotechnology Co Ltd. The enzyme-linked immunosorbent assay kit was used to detect the levels of interleukin-6 (IL-6) and C-reactive protein (CRP). Evaluation, instruct the patient to score the toothache in the past 24 hours according to their own subjective feelings and combined with the scale, with a total score of 0 to 10 points. The higher the score, the higher the pain, and the average score is calculated.

The article "Efficacy of Periodontal Endodontics Combined with Diode Laser (DL) Therapy on Severe Periodontitis" was retracted in 2023. Reasons: signs of a paper mill; suspected computer-generated content; unreliable results or conclusions; lack of ethics approval or compliance.

### 2.4. Statistical Analysis

All statistical data in this study were entered into Excel software by the first author and the corresponding author, and the statistical processing software was SPSS25.0 for calculation. Repeated measure analysis of variance between groups was used to measure the measurement which was expressed as mean ± standard deviation (*X* ± SD). Material. One-way analysis of variance was used for comparison between groups, and the count data were tested by *x*^2^. Count data expressed as a percentage (%) were tested by *χ*^2^. The risk factors with significant differences were screened. Included data that did not conform to a normal distribution were described by M (QR), using the Mann–Whitney test. The statistical significance was *P* < 0.05.

## 3. Results

### 3.1. Comparison of General Clinical Data

The comparison of general data such as gender, age, number of carious tooth surfaces, number of bits, and body mass index of the two groups of patients did not have significant statistical differences by independent sample *t*-test and chi-square test (*P* > 0.05) (see Table 1).

### 3.2. Comparison of Clinical Efficacy

Before treatment, there was no significant difference in clinical efficacy between the two groups. After 3 months of treatment, the bleeding index (BI), plaque index (PLI), and periodontal probing depth (PD) of the treatment group were significantly lower than those of the control group, and the difference was statistically significant (*P* < 0.05). The attachment loss (AL) of the group was not significantly different from that of the control group (*P* > 0.05) (see Figure 1).

### 3.3. Comparison of Inflammatory Factor Levels

Before treatment, there was no significant difference in the levels of inflammatory factors between the two groups (*P* > 0.05). After 3 months of treatment, the levels of IL-6 and CRP in the treatment group were significantly lower than those in the control group, and the difference was statistically significant (*P* < 0.05) (see Figure 2).

### 3.4. Toothache Comparison

Before treatment, there was no significant difference in the levels of inflammatory factors between the two groups (*P* > 0.05). After 3 days of treatment, the VAS score of the treatment group was significantly lower than that of the control group, and the difference was statistically significant (*P* < 0.05) (see Figure 3).

The article "Efficacy of Periodontal Endodontics Combined with Diode Laser (DL) Therapy on Severe Periodontitis" was retracted in 2023. Reasons: signs of a paper mill; suspected computer-generated content; unreliable results or conclusions; lack of ethics approval or compliance.

## 4. Discussion

DL is one of the most popular new periodontal techniques, which is easy to operate and the laser fiber can reach areas that cannot be reached by traditional mechanical methods, and can work on affected teeth with anatomical abnormalities such as deep periodontal pockets, root bifurcations, and root surface depressions [14]. When the DL beam is irradiated to biological tissues, it can produce thermal, photochemical, and biostimulatory effects to accelerate the inflammatory absorption and improve local microcirculation at the lesion site, which has good periodontal treatment functions with the ability to sterilize, promote healing, reduce bleeding, and remove epithelium from periodontal pockets [15]. Therefore, laser therapy that is applied to the adjuvant treatment of periodontal diseases has attracted wide attention from scholars at home and abroad [16]. DL is a tissue-penetrating laser, mainly applied to soft tissues, and the heat generated has minimal effect on the roots of teeth, and the energy generated can be absorbed by endogenous chromophores, of which hemoglobin has the highest absorption rate and can play the best role within the blood environment [17]. DL has the advantages of small size, light weight, low cost, adjustable wavelength, and stable output power, and it has a very broad development prospect [18].

Our study found that after 3 months of treatment, the bleeding index (BI), plaque index (PLI), and periodontal probing depth (PD) of the treatment group were significantly lower than those of the control group, indicating that the application of DL treatment had a significant effect. The reasons are as follows: periodontitis is a chronic inflammatory disease caused by bacterial infection, and the removal of pathogenic bacteria in the periodontal pocket is an important part of the treatment of periodontitis [19]. When measured four weeks after the completion of basic periodontal treatment, the subgingival microbial flora will change, in which the number of periodontal pathogens is significantly reduced [20]. The microbiota recolonized long after basic treatment. The microbial structure was very different from that of mature dental plaque in a shorter period of time after treatment, but the microbial structure and mature dental plaque structure after a long time of treatment were largely the same except for a few bacteria [21–25]. But this microbial change must be controlled by regular subgingival scaling and root planing performed during supportive periodontal therapy [26]. The addition of laser irradiation at this critical stage of treatment can effectively improve periodontal healing, achieve deeper bacterial suppression, and hopefully prolong the interval between repairs [27]. In the treatment of soft tissue, the use of DL treatment has a bactericidal effect. Since DL cannot remove dental calculus, it is only used here as an auxiliary means to treat its bactericidal and detoxifying effects [28]. DL treatment applied to the blood-rich periodontal pocket can better absorb the laser beam, and the resulting thermal effect can cause immediate damage to the cell wall structure of Gram-negative bacteria, but basically does not damage the root surface [29]. Biostimulatory effects can reduce vascular permeability, reduce inflammation, reduce congestion and edema, improve tissue blood circulation, promote angiogenesis and stimulate tissue regeneration, and are inexpensive, small, and simple to operate [30].

The article "Efficacy of Periodontal Endodontics Combined with Diode Laser (DL) Therapy on Severe Periodontitis" was retracted in 2023. Reasons: signs of a paper mill; suspected computer-generated content; unreliable results or conclusions; lack of ethics approval or compliance.

In our study, we found that IL-6 and CRP in the treatment group were significantly lower than those in the control group after 3 months of treatment, suggesting that DL treatment can effectively control the inflammatory response of the organism and improve the condition. The reasons are as follows: DL is currently a more common type of laser in oral diseases, which can be highly absorbed by water and water-rich tissues, producing a photothermal effect with less thermal damage compared to other lasers [31]. It is able to achieve a low thermal effect treatment and exerts a more refined effect of plaque and tartar removal [32]. It also stimulates fibroblasts, promotes the synthesis of collagen and extracellular matrix on the root surface, improves their biocompatibility, and provides good conditions for fibroblast attachment [33]. Also, the ability to remove the staining layer of the tooth surface in the bifurcation zone and promote the regeneration of periodontal tissues can further confirm that the combined treatment can enhance clinical efficacy and promote gingival health [34]. The pathological process of periodontitis is accompanied by the release of several inflammatory factors, which can be used for the evaluation of the disease [35]. IL-6 induces a variety of inflammatory responses and is able to inhibit the production of several periodontal membrane cells [36]. When subjected to microbial invasion, the nonspecific immune mechanisms of the body are activated and hepatocytes increase the synthesis of CRP [37]. CRP can bind to ligands to activate the complement and mononuclear phagocyte systems, enhancing the ability to undergo external microorganisms [38].

The article "Efficacy of Periodontal Endodontics Combined with Diode Laser (DL) Therapy on Severe Periodontitis" was retracted in 2023. Reasons: signs of a paper mill; suspected computer-generated content; unreliable results or conclusions; lack of ethics approval or compliance.

In our study, we found that the VAS scores of the treatment group were significantly lower than those of the control group after 3 d of treatment, indicating that the combined treatment was effective in improving the toothache and achieving significant therapeutic effects. Laser removal of diseased tissues by periodontal reversal, combined with laser to promote periodontal tissue repair, can achieve a strong therapeutic effect through continuous treatment, effectively relieving toothache and enhancing the therapeutic effect [39]. Inflammation of periodontal tissue in teeth with severe periodontitis can affect the pulp tissue and can lead to loss of attachment and irreducible inflammatory changes in the pulp or even necrosis [40]. Timely and complete DL treatment of teeth with severe periodontitis with sluggish pulp vitality can control the progression of inflammation and facilitate periodontal tissue healing [41]. Few studies have tracked the long-term prognosis of teeth with severe periodontitis after DL treatment, and further follow-up studies are needed in the future to determine the long-term efficacy of treatment [42]. However, the present study has some clinical implications, as most of the teeth with severe periodontitis with sluggish pulp vitality already have some degree of pulp degeneration or necrosis [43]. Patient's pain, and is also in line with the principle of minimally invasive treatment in the broad sense [44]. It is also in line with the principle of minimally invasive treatment in the broad sense [45].

Our study has certain limitations which are as follows: lack of long-termfollow-up, no observation of patients' recurrence, and our study does not meet the needs of multifaceted and multilevel observation of clinical trials. In conclusion, the application of DL treatment is effective in promoting periodontal tissue healing and reducing the depth of periodontal pockets, reducing the degree of tooth pain, and thus providing a reference for clinical treatment.

## Figures and Tables

**Figure 1:** Clinical efficacy comparison (all statistical clinical efficacy comparison data in this study were entered into Excel software by the first author and corresponding author, and the statistical processing software was SPSS25.0 for calculation. An independent sample t-test analysis was performed between the two groups to measure the values which were expressed as mean ± standard deviation. It was found that before treatment, there was no significant difference in clinical efficacy between the two groups. After 3 months of treatment, the bleeding index (BI), plaque index (PLI), and periodontal probing depth (PD) were significantly lower than those in the control group, and the difference was statistically significant (*P* < 0.05), while the attachment loss (AL) in the treatment group was not significantly different from that in the control group (*P* < 0.05).

The article "Efficacy of Periodontal Endodontics Combined with Diode Laser (DL) Therapy on Severe Periodontitis" was retracted in 2023. Reasons: signs of a paper mill; suspected computer-generated content; unreliable results or conclusions; lack of ethics approval or compliance.

**Figure 2:** Comparison of inflammatory factor levels (all statistical inflammatory factor level comparison data in this study were entered into Excel software by the first author and corresponding author, and the statistical processing software was SPSS25.0 for calculation. An independent sample t-test analysis was performed between the two groups to measure the measured values which were expressed as mean ± standard deviation. It was found that there was no significant difference in the levels of inflammatory factors between the two groups before treatment (*P* > 0.05). After 3 months of treatment, the levels of IL-6 and CRP in the treatment group were significantly lower than those in the control group, and the difference was statistically significant (*P* < 0.05).

**Figure 3:** Toothache degree comparison (all statistical toothache degree comparison data in this study were entered into Excel software by the first author and corresponding author, and the statistical processing software was SPSS25.0 for calculation. An independent sample *t*-test analysis was performed between the two groups to measure the measured values which were expressed as mean ± standard deviation. It was found that before treatment, there was no significant difference in the levels of inflammatory factors between the two groups (*P* > 0.05). The VAS score was significantly lower than that of the control group, and the difference was statistically significant (*P* < 0.05).

**Table 1:** Comparison of clinical data between two groups of patients (*n*, $\bar{x}\pm s$).

Clinical parameter	Comparison group (50)	Treatment group (50)	*χ * ^2^ * /t*	*P*
Sex (male/female)	23/27	24/26	0.040	0.841
Age (years)	56.13 ± 6.32	55.91 ± 6.67	0.169	0.866
Number of decayed tooth surfaces	44.78 ± 3.32	44.34 ± 3.25	0.670	0.505
Number of digits	123.62 ± 10.66	123.26 ± 10.64	0.169	0.866
Body mass index (kg/m^2^)	26.78 ± 2.32	26.94 ± 2.25	0.350	0.727

## Data Availability

No data were used to support this study.

## References

[1] Theodoro L. H., Marcantonio R. A. C., Wainwright M., Garcia V. G. (2021). LASER in periodontal treatment: is it an effective treatment or science fiction?. *Brazilian Oral Research*.

[2] Zheng L., Kang J. (2011). Evaluation of 6-year maintenance effect of periodontal non-surgical treatment of a case of chronic periodontitis with deformed radicular groove. *Journal of West China Journal of Stomatology*.

[3] Tan B., Xiao J., Wu W. Application of root canal therapy in the treatment of recurrent periodontal abscess.

The article "Efficacy of Periodontal Endodontics Combined with Diode Laser (DL) Therapy on Severe Periodontitis" was retracted in 2023. Reasons: signs of a paper mill; suspected computer-generated content; unreliable results or conclusions; lack of ethics approval or compliance.

[4] Zhang X., Sun C., Xue C. (2013). Semiconductor diode laser and its application in periodontal surgery. *Chinese Journal of Practical Stomatology*.

[5] Li Y., Wang X., Xu J., Zhou X., Xie K. (2012). The clinical study on the use of diode laser irradiation in the treatment of periodontal-endodontic combined lesions. *West China Journal of Stomatology*.

[6] Giannelli M., Materassi F., Fossi T., Lorenzini L., Bani D. (2018). Treatment of severe periodontitis with a laser and light-emitting diode (LED) procedure adjunctive to scaling and root planing: a double-blind, randomized, single-center, split-mouth clinical trial investigating its efficacy and patient-reported outcomes at 1 year. *Lasers in Medical Science*.

[7] Katsikanis F., Strakas D., Vouros I. (2020). The application of antimicrobial photodynamic therapy (aPDT, 670 nm) and diode laser (940 nm) as adjunctive approach in the conventional cause-related treatment of chronic periodontal disease: a randomized controlled split-mouth clinical trial. *Clinical Oral Investigations*.

[8] Chandra S., Shashikumar P. (2018). Diode laser—a novel therapeutic approach in the treatment of chronic periodontitis in type 2 diabetes mellitus patients: a prospective randomized controlled clinical trial. *Journal of Lasers in Medical Sciences*.

[9] Kaplan T., Sezgin G. P., Sönmez Kaplan S. (2021). Effect of a 980-nm diode laser on post-operative pain after endodontic treatment in teeth with apical periodontitis: a randomized clinical trial. *BMC Oral Health*.

[10] Pourshahidi S., Ebrahimi H., Mansourian A., Mousavi Y., Kharazifard M. (2019). Comparison of Er, Cr: YSGG and diode laser effects on dentin hypersensitivity: a split-mouth randomized clinical trial. *Clinical Oral Investigations*.

[11] Crispino A., Figliuzzi M. M., Iovane C. (2015). Effectiveness of a diode laser in addition to non-surgical periodontal therapy: study of intervention. *Annali di Stomatologia*.

[12] Lobo T. M., Pol D. G. (2015). Evaluation of the use of a 940 nm diode laser as an adjunct in flap surgery for treatment of chronic periodontitis. *Journal of Indian Society of Periodontology*.

[13] Meng H. (2019). An introduction to the new international classification of periodontal disease and peri-implant disease in 2018. *Journal of Chinese Journal of Stomatology.*.

[14] Chambrone L., Ramos U. D., Reynolds M. A. (2018). Infrared lasers for the treatment of moderate to severe periodontitis: an American Academy of periodontology best evidence review. *Journal of Periodontology*.

[15] Cherepynska Y., Volkova O., Riabokon E., Baglyk T. (2017). Analysis of the long-term clinical results of using 940 *μ*m diode laser in patients with generalized moderate chronic periodontitis. *Georgian Med News*.

The article "Efficacy of Periodontal Endodontics Combined with Diode Laser (DL) Therapy on Severe Periodontitis" was retracted in 2023. Reasons: signs of a paper mill; suspected computer-generated content; unreliable results or conclusions; lack of ethics approval or compliance.

[16] Jokar L., Bayani M., Hamidi H., Keivan M., Azari-Marhabi S. (2019). A comparison of 940 nm diode laser and cryosurgery with liquid nitrogen in the treatment of gingival physiologic hyperpigmentation using split mouth technique: 12 months follow up. *Journal of Lasers in Medical Sciences*.

[17] Yang C., Wang X., Wang Y. (2022). Effect of diode laser combined with minocycline hydrochloride in nonsurgical periodontal therapy: a randomized clinical trial. *BMC Oral Health*.

[18] Shahnaz A., Jamali R., Mohammadi F., Khorsand A., Moslemi N., Fekrazad R. (2018). A preliminary randomized clinical trial comparing diode laser and scalpel periosteal incision during implant surgery: impact on postoperative morbidity and implant survival. *Lasers in Medical Science*.

[19] Giannelli M., Formigli L., Bani D. (2014). Comparative evaluation of photoablative efficacy of erbium: yttrium-aluminium-garnet and diode laser for the treatment of gingival hyperpigmentation. A randomized split-mouth clinical trial. *Journal of Periodontology*.

[20] Castro G. L., Gallas M., Núñez I. R., Borrajo J. L. L., Garcíavarela L. (2006). Histological evaluation of the use of diode laser as an adjunct to traditional periodontal treatment. *Photomedicine and Laser Surgery*.

[21] Sanz-Moliner J. D., Nart J., Cohen R. E., Ciancio S. G. (2013). The effect of an 810-nm diode laser on postoperative pain and tissue response after modified Widman flap surgery: a pilot study in humans. *Journal of Periodontology*.

[22] Ciurescu C. E., Gutknecht N., Ciurescu V. A. (2021). Two-year outcomes following the adjunctive use of InGaAsP and Er, Cr:YSGG lasers in nonsurgical periodontal therapy in patients with stages III and IV periodontitis. *Quintessence International*.

[23] Bassir S. H., Moslemi N., Jamali R. (2013). Photoactivated disinfection using light-emitting diode as an adjunct in the management of chronic periodontitis: a pilot double-blindsplit-mouth randomized clinical trial. *Journal of Clinical Periodontology*.

[24] Dureja D., Sharma H., Agarwal M., Srivastava S., Tandon P. (2020). Hereditary gingival fibromatosis: a report of a rare case in siblings and its management using diode laser. *Contemporary Clinical Dentistry*.

[25] Campos L., Gallottini M., Pallos D., Simões A., Martins F. (2018). High-power diode laser on management of drug-induced gingival overgrowth: report of two cases and long-termfollow-up. *Journal of Cosmetic and Laser Therapy*.

[26] Roncati M. (2021). Impact of home and professional care on laser-assisted management of peri-implant complications: a case report. *The International Journal of Periodontics and Restorative Dentistry*.

The article "Efficacy of Periodontal Endodontics Combined with Diode Laser (DL) Therapy on Severe Periodontitis" was retracted in 2023. Reasons: signs of a paper mill; suspected computer-generated content; unreliable results or conclusions; lack of ethics approval or compliance.

[27] Wang P., Zhang H., Chen D. (2011). Detection and analysis of nickel and chromium elements in blood and urine of patients after nickel-chromium alloy porcelain crown repair. *Journal of Hebei Medicine*.

[28] Xu B., Wang X., Song J. Investigation of urinary nickel and chromium levels in patients with nickel-chromium porcelain crown restoration.

[29] Bishara S. E., Barrett R. D., Selim M. I. (1993). Biodegradation of orthodontic appliances. Part II. Changes in the blood level of nickel. *American Journal of Orthodontics and Dentofacial Orthopedics*.

[30] Jaikumar S., Srinivasan L., Kennedy Babu S. P. K., Gandhimadhi D., Margabandhu M. (2022). Laser-assisted frenectomy followed by post-operative tongue exercises in ankyloglossia: a report of two cases. *Cureus*.

[31] Ozberk S. S., Gündoğar H., Şenyurt S. Z., Erciyas K. (2017). Adjunct use of low-level laser therapy on the treatment of necrotizing ulcerative gingivitis: a case report. *Journal of Lasers in Medical Sciences*.

[32] de Oliveira Guaré R., Costa S. C., Baeder F., de Souza Merli L. A., Dos Santos M. T. B. R. (2010). Drug-induced gingival enlargement: biofilm control and surgical therapy with gallium-aluminum-arsenide (GaAlAs) diode laser-A2-yearfollow-up. *Special Care in Dentistry*.

[33] Annaji S., Sarkar I., Rajan P. (2016). Efficacy of photodynamic therapy and lasers as an adjunct to scaling and root planing in the treatment of aggressive periodontitis—a clinical and microbiologic short term study. *Journal of Clinical and Diagnostic Research*.

[34] Devi P. K., Kumar G. P., Bai Y. D., Ammaji A. D. (2013). Ipsilateral idiopathic gingival enlargement and it’s management using conventional gingivectomy and diode laser: a recurrent case after 15 years. *Journal of Indian Society of Periodontology*.

[35] Silva L. A. B., Novaes A. B., de Oliveira R. R., Nelson-Filho P., Santamaria M., Silva R. A. B. (2012). Antimicrobial photodynamic therapy for the treatment of teeth with apical periodontitis: a histopathological evaluation. *Journal of Endodontics*.

[36] Del Giudice M., Gangestad S. W. (2018). Rethinking IL-6 and CRP: why they are more than inflammatory biomarkers, and why it matters. *Brain, Behavior, and Immunity*.

[37] Beavers D. P., Kritchevsky S. B., Gill T. M. (2021). Elevated IL-6 and CRP levels are associated with incident self-reported major mobility disability: a pooled analysis of older adults with slow gait speed. *The Journals of Gerontology: Series A*.

[38] Ridker P. M., Rane M. (2021). Interleukin-6 signaling and anti-interleukin-6 therapeutics in cardiovascular disease. *Circulation Research*.

The article "Efficacy of Periodontal Endodontics Combined with Diode Laser (DL) Therapy on Severe Periodontitis" was retracted in 2023. Reasons: signs of a paper mill; suspected computer-generated content; unreliable results or conclusions; lack of ethics approval or compliance.

[39] Roncati M., Gariffo A. (2016). Three years of a nonsurgical periodontal treatment protocol to observe clinical outcomes in ≥6-mm pockets: a retrospective case series. *The International Journal of Periodontics and Restorative Dentistry*.

[40] Martins S. H. L., Novaes A. B., Taba M. (2017). Effect of surgical periodontal treatment associated to antimicrobial photodynamic therapy on chronic periodontitis: a randomized controlled clinical trial. *Journal of Clinical Periodontology*.

[41] Azaripour A., Azaripour M., Willershausen I., Noorden C. J. F. V., Willershausen B. (2018). Photodynamic therapy has no adverse effects *in vitro* on human gingival fibroblasts and osteoblasts. *Clinical Laboratory*.

[42] Kreisler M., Al Haj H., Daubländer M. (2002). Effect of diode laser irradiation on root surfaces *in vitro*. *Journal of Clinical Laser Medicine and Surgery*.

[43] Salavadhi S. S., Chintalapani S., Ramachandran R., Nagubandi K., Ramisetti A., Boyapati R. (2017). Atomic force microscopy: a three-dimensional reconstructive tool of oral microbiota in gingivitis and periodontitis. *Journal of Indian Society of Periodontology*.

[44] Gomes M. F., Goulart M. D. G. V., Giannasi L. C. (2018). Effects of the photobiomodulation using different energy densities on the periodontal tissues under orthodontic force in rats with type 2 diabetes mellitus. *Brazilian Oral Research*.

[45] Schwarz F., Sculean A., Berakdar M., Szathmari L., Georg T., Becker J. (2003). *In vivo* and *in vitro* effects of an Er:YAG laser, a GaAlAs diode laser, and scaling and root planing on periodontally diseased root surfaces: a comparative histologic study. *Lasers in Surgery and Medicine*.

